# External Mechanical Work and Pendular Energy Transduction of Overground and Treadmill Walking in Adolescents with Unilateral Cerebral Palsy

**DOI:** 10.3389/fphys.2016.00121

**Published:** 2016-04-13

**Authors:** Marie Zollinger, Francis Degache, Gabriel Currat, Ludmila Pochon, Nicolas Peyrot, Christopher J. Newman, Davide Malatesta

**Affiliations:** ^1^Institute of Sport Sciences of University of Lausanne, University of LausanneLausanne, Switzerland; ^2^Health Research Unit, School of Health Sciences, University of Applied Sciences Western SwitzerlandLausanne, Switzerland; ^3^IRISSE Laboratory (EA4075), UFR SHE, University of La RéunionLe Tampon, France; ^4^Pediatric Neurology and Neurorehabilitation Unit, Lausanne University HospitalLausanne, Switzerland; ^5^Department of Physiology, Faculty of Biology and Medicine, University of LausanneLausanne, Switzerland

**Keywords:** biomechanics, gait, human locomotion, inverted pendulum, exercise

## Abstract

**Purpose:** Motor impairments affect functional abilities and gait in children and adolescents with cerebral palsy (CP). Improving their walking is an essential objective of treatment, and the use of a treadmill for gait analysis and training could offer several advantages in adolescents with CP. However, there is a controversy regarding the similarity between treadmill and overground walking both for gait analysis and training in children and adolescents. The aim of this study was to compare the external mechanical work and pendular energy transduction of these two types of gait modalities at standard and preferred walking speeds in adolescents with unilateral cerebral palsy (UCP) and typically developing (TD) adolescents matched on age, height and body mass.

**Methods:** Spatiotemporal parameters, external mechanical work and pendular energy transduction of walking were computed using two inertial sensors equipped with a triaxial accelerometer and gyroscope and compared in 10 UCP (14.2 ± 1.7 year) and 10 TD (14.1 ± 1.9 year) adolescents during treadmill and overground walking at standard and preferred speeds.

**Results:** The treadmill induced almost identical mechanical changes to overground walking in TD adolescents and those with UCP, with the exception of potential and kinetic vertical and lateral mechanical works, which are both significantly increased in the overground-treadmill transition only in UCP (*P* < 0.05).

**Conclusions:** Adolescents with UCP have a reduced adaptive capacity in absorbing and decelerating the speed created by a treadmill (i.e., dynamic stability) compared to TD adolescents. This may have an important implication in rehabilitation programs that assess and train gait by using a treadmill in adolescents with UCP.

## Introduction

Walking impairments associated with neuromuscular weakness and low aerobic fitness may be involved in chronic fatigue and induce important limitations in the daily walking activity of children and adolescents with cerebral palsy (CP) compared with typically developing (TD) children and adolescents (Brunton and Rice, 2012). One of the aims of therapeutic interventions is to help these patients achieve maximal independence by improving their functional capacity and mobility (Myrhaug et al., 2014). To improve their walking is an essential objective and the use of a treadmill for walking analysis and training may offer several advantages, such as the opportunity to repeat and train the gait cycle at controlled and fixed walking speeds. Moreover, it has been suggested that treadmill training is safe, feasible and effective for children and adolescents with CP, especially for those with balance disorders (Willoughby et al., 2009).

There is a controversy regarding the similarity between treadmill and overground walking both in gait analysis and in the effective transfer to overground walking of the locomotor adaptations obtained after treadmill training (i.e., functional adaptation). The visual-kinaesthetic conflict during treadmill walking implies a recalibration of the motor output and a higher “neuronal-computational” effort (Zanetti and Schieppati, 2007). Recent evidence has indicated that similar neural networks may be involved in treadmill and overground walking (Choi and Bastian, 2007) and that there are only minor kinetic and spatiotemporal changes between these modalities for any given speed in healthy adults and children (i.e., a slightly increased step frequency and shorter step length <10% on treadmill, Stolze et al., 1997; Warabi et al., 2005; Lee and Hidler, 2008).

Only two studies compared spatiotemporal parameters during treadmill and overground walking in children with unilateral cerebral palsy (Matsuno et al., 2010; van der Krogt et al., 2014). These studies showed that their preferred walking speed (PWS) was slower with a slower step frequency, a shorter step length and stance duration on treadmill compared with overground walking. These spatiotemporal changes were similar in children with CP and TD children, attesting that the treadmill induced similar locomotor adaptations in the two groups and that this tool can be considered useful to highlight and study gait deviations and fatigue effects during walking in patients with CP (van der Krogt et al., 2014). However, the comparison of biomechanical variables of gait for the two walking conditions, each at a different speed, represented a methodological limitation. In order to isolate the effect of the walking condition on the gait pattern, it is important to compare both conditions at the same speed (i.e., standard walking speed, SWS) and to use the assessment of the PWS to investigate “gait behavioral adaptations” (Hortobagyi et al., 2011) in both walking conditions. Recently, (van der Krogt et al., 2015) compared kinetics of the two walking conditions in children with CP and showed that, in treadmill compared to overground gait, there was a shift from an ankle to a hip strategy, with lower ankle power generation and absorption and increased hip moment and work, likely due to a backward positioning of the hip and a more forward trunk lean. As previously suggested (van der Krogt et al., 2015), this gait strategy change may contribute to increase energy cost and thus mechanical work of walking in children with CP (Donelan et al., 2002a). In fact, total mechanical work (*W*_*tot*_) is higher in CP than in TD during overground walking (Olney et al., 1987; van den Hecke et al., 2007). This greater *W*_*tot*_ is associated with higher internal mechanical work (*W*_*int*_: the work associated with the acceleration of body segments with respect to the body mass center, COM) and external mechanical work (*W*_*ext*_: the work performed by the muscles to translate the COM with respect to the ground; Cavagna and Kaneko, 1977). The latter depends on pendular transduction of potential into kinetic energy, due to the vertical shift of the COM and its forward speed, respectively (Cavagna and Kaneko, 1977). This pendular energy transduction (i.e., inverted pendulum recovery of mechanical energy of the COM), a summary indicator for the mechanics of pathological gait (Detrembleur et al., 2000), is impaired in children with CP (Olney et al., 1987; van den Hecke et al., 2007). To the best of our knowledge, no studies have been conducted to compare external mechanical work and pendular energy transduction of overground and treadmill walking in CP adolescents, in order to determine whether the treadmill could be a useful tool for clinical gait analysis and as an adequate alternative to overground walking assessment in this population.

Therefore, the aim of our study was to compare the external mechanical work and pendular energy transduction of overground and treadmill walking at SWS and PWS in unilateral CP and TD adolescents matched on age, height and body mass. We hypothesized that after acclimation treadmill walking compared with overground walking would induce similar mechanical changes at SWS. However, at this speed in both gait modalities, *W*_*ext*_ should be higher in adolescents with CP than in TD adolescents. We also examined the hypothesis that PWS would be faster overground in both groups compared to treadmill walking, and that for the two gait modalities the slower PWS in adolescents with CP would be associated with similar or higher *W*_*ext*_ as compared to TD adolescents.

## Materials and methods

### Participants

A convenience sample of 10 adolescents with unilateral spastic cerebral palsy (UCP, 14.2 ± 1.7 year) and 10 typically developing adolescents (TD, 14.1 ± 1.9 year) participated in this study. The UCP adolescents were recruited from the outpatient clinic of the Pediatric Neurology and Neurorehabilitation Unit, Lausanne University Hospital. Inclusion criteria were (1) age 10–16 years; (2) unilateral spastic CP diagnosed by a pediatric neurologist and/or physiatrist; (3) low level of spasticity (Ashworth 1 and 2; Ashworth, 1964); (4) level I or II of the Gross Motor Function Classification System (GMFCS) (Palisano et al., 1997); (5) cognitive ability to understand instructions. The TD group was recruited via an e-mail to collaborators of the Unit and selected on age, height and body mass matching the UCP population. Exclusion criteria for both groups were mental retardation or severe learning difficulties and severe visual disorders. The local ethics committee approved the study protocol and the participants and their parents approved and signed the informed written consent. Each participant received a bookshop voucher for their participation.

### Experimental design

Each adolescent completed one test session at the Pediatric Neurology and Neurorehabilitation Unit. After a brief introduction to the experimental procedures for the participants and their parents, the anthropometric characteristics of adolescents were assessed. Then, overground and treadmill gait pattern assessments were performed during walking in shoes. For overground walking measurements, the adolescents were asked to walk on a 30-m walkway at PWS and SWS (i.e., 3.5 km.h^−1^, the average PWS of UCP adolescents reported in the literature, Marconi et al., 2014). For SWS, all participants followed a technician, placed on their left side, who walked at a constant speed paced by a portable MP3 player, with an audio feedback (i.e., one beep every 2 m). For the treadmill gait pattern evaluation, after 10 min of treadmill accommodation (Matsas et al., 2000) across different walking speeds (1–5 km.h^−1^) and a brief rest period, the PWS of the participants was determined according to the procedure previously described by Martin et al. (1992). Then, the participants were asked to walk at PWS and SWS (3.5 km.h^−1^). For each walking speed and condition, ten consecutive strides were collected and selected for biomechanical analysis.

### Assessments and data analysis

#### Anthropometric measurements

Standing height was measured using a Harpenden stadiometer. Body mass was measured to the nearest 0.1 kg on a precision digital scale with the subject wearing shorts and a T-shirt.

#### Gait pattern

Mechanical parameters of walking were assessed from the three-dimensional accelerations of two inertial sensors equipped with a triaxial (three orthogonal axes) accelerometer and gyroscope (MTx, Xsens, Enshede, The Netherlands). According to Peyrot et al. (2009, 2010) the first sensor was taped and secured directly to the skin on the lower part of the back, facing the L3 vertebra region (close to COM), using an adhesive strap and was used to measure the COM accelerations. The other inertial/gyroscope sensor, used to measure the three dimensional accelerations of the foot, was also taped and secured on the instep of subjects non-paretic limb for UCP and on the instep of the dominant limb for TD. The non-paretic limb was chosen for adolescents with UCP since it has been shown that the asymmetry in gait profile score is similar on the affected and unaffected side in GMFCS level I and II unilateral adolescents with CP (Lundh et al., 2014; see the paragraph “Methodological limitations” in the Discussion). As described in detail by Pfau et al. (2005), the orientation algorithm of the inertial sensors provided orientation data in the earth reference system (horizontal and magnetic north) in the form of Euler angles (roll, pitch, and heading). Euler angles represent rotations of the sensor system into the earth reference system, with the magnetic north corresponding to the antero-posterior axis in our study. Thus, rotation matrices were used to reposition three-dimensional accelerations of the two sensors in the earth reference system. Data were recorded at a sample rate of 100 Hz and low-pass filtered at 30 Hz (fourth-order, zero-lag, low-pass Butterworth).

#### Spatiotemporal parameters

Spatiotemporal parameters were measured with the inertial sensor located on the instep of the foot of the subject. As described by Jasiewicz et al. (2006), heel strike and toe-off were determined from forward and vertical foot acceleration peaks. The stride duration (delimited by two consecutive heel strikes) and stance duration (heel strike to consecutive toe-off) were computed, as well as single support duration of the contralateral limb (toe-off to heel strike of the foot equipped). Then, the stance and single support durations were expressed relative to stride duration (%). The stride frequency (Hz) was computed as the inverse of stride duration, and stride length as walking speed divided by stride frequency (Peyrot et al., 2010).

#### External mechanical work and potential-kinetic energy transduction

As previously described (Peyrot et al., 2009, 2010), the inertial sensors located on the lower part of the back permitted the computation of kinetic aspects of walking related to the displacement of the COM (Pfau et al., 2005; Meichtry et al., 2007). The three-dimensional accelerations of the COM determined the vertical, forward, and medio-lateral COM accelerations and the external mechanical work (*W*_*ext*_) was calculated, as previously proposed (Cavagna, 1975). Integrations were used to determine the COM velocity and displacement in the three directions. The instantaneous potential energy of the COM (*E*_*p*_; J) was computed from vertical displacement (*h; m*), body mass (*m*; kg), and gravitational constant (*g:* 9.81 m.s^−2^; Equation 1). From the instantaneous vertical (*V*_*y*_; m.s^−1^), horizontal (*V*_*x*_; m.s^−1^), and lateral (*V*_*z*_; m.s^−1^) velocities and *m*, the instantaneous total (*E*_*k*_; J), vertical (*E*_*kv*_; J), forward (*E*_*kf*_; J), and lateral (*E*_*kl*_; J) kinetic energy of the COM were computed (Equation 2).

(1) $$\begin{array}{l} E_{p}=mgh \end{array}$$

(2) $$\begin{array}{l} E_{k}=E_{kv}+E_{kf}+E_{kl}=0.5m\left[{\left(V_{y}\right)}^{2}+{\left(V_{x}\right)}^{2}+{\left(V_{z}\right)}^{2}\right] \end{array}$$

The total mechanical energy of the COM (*E*_*tot*_; J) was calculated as the sum of *E*_*k*_ and *E*_*p*_ and the external mechanical work (*W*_*ext*_, J) as the sum of the positive increments in *E*_*tot*_, and divided by stride length and the body mass of the subject to be expressed in J.kg^−1.^m^−1^. The same procedure was applied to calculate total (*W*_*k*_), vertical (*W*_*kv*_), forward (*W*_*kf*_), lateral (*W*_*kl*_) kinetic mechanical work, and potential mechanical work (*W*_*p*_), as the sum of the positives increments in respective energies (Peyrot et al., 2009, 2010).

The inverted pendulum recovery of mechanical energy of the COM (*R*; %) was calculated (Peyrot et al., 2009; Equation 3).

(3) $$\begin{array}{l} R=\frac{W_{k}+W_{p}-W_{ext}}{W_{k}+W_{p}}\times 100 \end{array}$$

The magnitude of *W*_*ext*_ and *R* depends on the relative magnitude of *W*_*k*_ and *W*_*p*_ (i.e., *W*_*k*_/*W*_*p*_) and phase shifts (α and β) of the fluctuations in *E*_*k*_ and *E*_*p*_ (Malatesta et al., 2009; Equations 4, 5, respectively).

(4) $$\begin{array}{r} \alpha =360^{{}^{\circ}}\frac{t_{pk+}}{\tau } \end{array}$$

(5) $$\begin{array}{r} \beta =360^{{}^{\circ}}\frac{t_{pk-}}{\tau } \end{array}$$

where τ is the step period; *T*_*pk*+_, period when *E*_*k*_ and *E*_*p*_ increase simultaneously; *T*_*pk*−_, period when *E*_*k*_ and *E*_*p*_ decrease simultaneously. Given this definition of α and β, if *E*_*k*_ and *E*_*p*_ fluctuated 180° out of phase, α and β would be equal to 0° (Cavagna et al., 2002).

The lateral COM displacement was equal to the total amplitude (from left to right) of the lateral COM position computed by integration of the lateral velocity over the mean stride (Peyrot et al., 2009, 2010).

### Statistical analysis

Data are expressed as means ± SD for all variables. A *t*-test was used to test differences between anthropometric characteristics of the two groups. For each walking speed (i.e., SWS and PWS) a 2-way repeated-measures mixed design ANOVA [condition (treadmill vs. overground) × group (UCP vs. TD)] followed by contrasts was used to determine the effects of the two walking conditions on biomechanical parameters in the two groups. The level of significance was set at *P* ≤ 0.05.

## Results

### Participants

The anthropometric characteristics of the study participants are presented in the Table 1. Nine adolescents with UCP were classified as GMFCS level I and 1 as GMFCS level II.

**Table 1:** **Participants characteristics**.

**Variable**	**UCP (*n* = 10)**	**TD (*n* = 10)**	***P*-value**
Boys/Girls	3/7	1/9	−
Age (years)	14.2 ± 1.7	14.1 ± 1.9	0.88
Body mass (kg)	56.4 ± 14.1	46.1 ± 11.0	0.07
Height (cm)	161.4 ± 9.2	156.1 ± 12.3	0.29

*Mean values ± standard deviation (SD). UCP, unilateral cerebral palsy adolescents; TD, typically developing adolescents; n, number of participants*.

### Spatiotemporal parameters

#### Standard walking speed

Stride duration and length were significantly lower, whereas stride frequency was significantly higher, during treadmill compared to overground walking in both groups (*P* ≤ 0.009*;* Table 2). There were no significant differences in the single and double support durations between walking conditions and groups (*P* ≥ 0.2; Table 2). The lateral COM displacements were significantly higher in the overground condition compared to treadmill walking (*P* = 0.021) and in UCP compared with TD within both walking conditions (*P* < 0.001; Table 2).

**Table 2:** **Spatiotemporal parameters at standard walking speed (SWS)**.

**Variable**	**UCP (*****n*** = **10)**		**TD (*****n*** = **10)**		***P*-value**
	**Overground**	**Treadmill**	**Overground**	**Treadmill**	
SWS, km^.^h^−1^	3.54 ± 0.06	3.50 ± 0.00	3.57 ± 0.07	3.50 ± 0.00	0.41
Stride duration, s	1.19 ± 0.04	1.12 ± 0.06	1.22 ± 0.05	1.15 ± 0.07	0.88^*^
Stride length, m	1.18 ± 0.04	1.09± 0.06	1.21 ± 0.06	1.11 ± 0.07	0.92^*^
Stride frequency, Hz	0.84 ± 0.03	0.90 ± 0.05	0.82 ± 0.03	0.87 ± 0.06	0.84^*^
Single support duration, %	74.5 ± 2.2	75.6 ± 1.7	76.6 ± 3.6	76.5 ± 2.9	0.15
Double support duration, %	25.5 ±2.2	24.4 ± 1.7	23.4 ± 3.6	23.5 ± 2.9	0.15
Lateral COM displacements, cm	4.7 ± 1.0	4.5 ± 0.6	3.5 ± 0.3	3.0 ± 0.6	0.31^*^^†^

*Mean values ± standard deviation (SD). n, number of participants; UCP, unilateral cerebral palsy adolescents; TD, typically developing adolescents; COM, center of mass; P-value, P value for interaction [condition (overground vs. treadmill) x group (UCP vs. TD)] of the 2-way repeated-measures mixed design ANOVA*.

* For significant condition (overground vs. treadmill) effect;

† *For significant group (UCP vs. TD) effect (P ≤ 0.05)*.

#### Preferred walking speed

PWS was significantly slower during treadmill walking compared with overground walking in both groups (*P* ≤ 0.001; Table 3). On the treadmill the stride length and frequency were significantly lower and the stride duration was significantly longer in both groups (*P* ≤ 0.001; Table 3), compared to overground walking. In treadmill walking the single support duration was significantly shorter (*P* = 0.001), whereas the double support duration was significantly longer (*P* = 0.001; Table 3), compared to overground walking. Only the lateral COM displacements showed a significant interaction effect and were significantly higher in treadmill than in overground walking (*P* < 0.001) and in UCP compared with TD within both walking conditions (*P* < 0.001; Table 3).

**Table 3:** **Spatiotemporal parameters at preferred walking speed (PWS)**.

**Variable**	**UCP (*****n*** = **9)**		**TD (*****n*** = **10)**		***P*-value**
	**Overground**	**Treadmill**	**Overground**	**Treadmill**	
PWS, km^.^h^−1^	4.28 ± 0.32	3.30 ± 0.32	4.76 ± 0.97	3.39 ± 0.68	0.27^*^
Stride duration, s	1.07 ± 0.04	1.16 ± 0.11	1.03 ± 0.12	1.16 ± 0.14	0.49^*^
Stride length, m	1.27 ± 0.07	1.06 ± 0.13	1.33 ± 0.16	1.08 ± 0.13	0.47^*^
Stride frequency, Hz	0.94 ± 0.04	0.87 ± 0.08	0.98 ± 0.11	0.87 ± 0.11	0.38^*^
Single support duration, %	77.0 ± 2.4	74.9 ± 2.0	79.2 ± 4.0	75.6 ± 3.3	0.34^*^
Double support duration, %	23.0 ± 2.4	25.1 ± 2.0	20.9 ± 4.0	24.4 ± 3.3	0.34^*^
Lateral COM displacements, cm	3.8 ± 0.5	4.9 ± 0.7	2.6 ± 0.4	3.0 ± 0.6	0.04^*^^†^

*Mean values ± standard deviation (SD). n, number of participants; UCP, unilateral cerebral palsy adolescents; TD, typically developing adolescents; COM, center of mass; P-value, P value for interaction [condition (overground vs. treadmill) x group (UCP vs. TD)] of the 2-way repeated-measures mixed design ANOVA*.

* For significant condition (overground vs. treadmill) effect;

† *For significant group (UCP vs. TD) effect (P ≤ 0.05)*.

### External mechanical work and potential-kinetic energy transduction

#### Standard walking speed

As shown in Table 4, *W*_*ext*_ was significantly higher on the treadmill compared with overground walking (*P* ≤ 0.012; Figure 1A) and in UCP compared with TD (*P* ≤ 0.027). *R* was significantly lower during treadmill than during overground walking in both groups (*P* = 0.001). There was no significant walking condition effect for *W*_*p*_ (*P* = 0.36; Figure 1B), β (*P* = 0.12), and *W*_*k*_/*W*_*p*_ (*P* = 0.76). However, *W*_*p*_ and β were significantly higher (*P* ≤ 0.003 and *P* ≤ 0.041, respectively) and *W*_*k*_/*W*_*p*_ was significantly lower (*P* ≤ 0.012) in UCP than in TD during treadmill and overground walking. *W*_*kv*_ and *W*_*kl*_ showed a significant interaction effect and were significantly higher in treadmill than in overground walking (*P* ≤ 0.002; Figures 1C,D) and in UCP compared with TD within both walking conditions (*P* ≤ 0.01). There were no significant differences in *W*_*k*_*, W*_*kf*_ and α between walking conditions and groups (*P* ≥ 0.17).

**Table 4:** **External mechanical work and potential-kinetic energy transduction at standard walking speed (SWS)**.

**Variable**	**UCP (*****n*** = **10)**		**TD (*****n*** = **10)**		***P*-value**
	**Overground**	**Treadmill**	**Overground**	**Treadmill**	
*W_*ext*_*, J·kg^−1.^m^−1^	0.44 ± 0.09	0.49 ± 0.13	0.36 ± 0.06	0.39 ± 0.05	0.38^*^^†^
*W_*p*_*, J·kg^−1.^m^−1^	0.56 ± 0.08	0.60 ± 0.09	0.46 ± 0.08	0.45 ± 0.10	0.10^†^
*W_*k*_*, J·kg^−1.^m^−1^	0.66 ± 0.09	0.66 ± 0.16	0.63 ± 0.10	0.62 ± 0.08	0.69
*W_*kf*_*, J·kg^−1.^m^−1^	0.64 ± 0.09	0.63 ± 0.15	0.61 ± 0.09	0.60 ± 0.08	0.99
*W_*kv*_*, J·kg^−1.^m^−1^	0.07 ± 0.02	0.09 ± 0.02	0.04 ± 0.01	0.05 ± 0.01	0.014^*^^†^
*W_*kl*_*, J·kg^−1.^m^−1^	0.04 ± 0.02	0.05 ± 0.02	0.02 ± 0.00	0.02 ± 0.00	0.002^*^^†^
*R*, %	64.2 ± 7.0	59.3 ± 8.1	66.5 ± 4.1	63.0 ± 5.6	0.53^*^
W_*k*_/W_*p*_	1.19 ± 0.23	1.10 ± 0.21	1.40 ± 0.26	1.46 ± 0.45	0.12^†^
α, °	24.2 ± 11.7	28.0 ± 10.1	23.1 ± 9.7	26.1 ± 12.2	0.85
β, °	23.1 ± 9.7	26.0 ± 10.7	13.7 ± 8.2	15.7 ± 10.3	0.73^†^

*Mean values ± standard deviation (SD). n, number of participants; UCP, unilateral cerebral palsy adolescents; TD, typically developing adolescents. W_ext_, external mechanical work; W_p_, potential mechanical work; W_k_, kinetic mechanical work; W_kf_, forward kinetic mechanical work; W_kv_, vertical kinetic mechanical work; W_kl_, lateral kinetic mechanical work; R, recovery; α, phase shift between the maximum of E_k_ and the minimum of E_p_; β, phase shift between the minimum of E_k_ and the maximum of E_p_; P-value, P value for interaction [condition (overground vs. treadmill) x group (UCP vs. TD)] of the 2-way repeated-measures mixed design ANOVA*.

* For significant condition (overground vs. treadmill) effect;

† *For significant group (UCP vs. TD) effect (P ≤ 0.05)*.

**Figure 1:** **External (A), potential (B), vertical kinetic (C), lateral kinetic (D) mechanical works at standard walking speed (SWS)**. UCP, unilateral cerebral palsy adolescents; TD, typically developing adolescents; OG, overground; TM, treadmill; *W*_*ext*_, external mechanical work; *W*_*p*_, potential mechanical work; *W*_*kv*_, vertical kinetic mechanical work; *W*_*kl*_, lateral kinetic mechanical work; ^*^For significant condition (overground vs. treadmill) effect;^†^For significant group (UCP vs. TD) effect;°For significant interaction (condition × group) effect (*P* ≤ 0.05).

#### Preferred walking speed

As shown in the Table 5, *W*_*k*_, *W*_*kf*_*, W*_*kv*_ (Figure 2C) and α were significantly lower in treadmill compared with overground walking in both groups (*P* ≤ 0.019). Similarly, *W*_*ext*_ tended to be lower in treadmill than in overground walking in UCP and TD (*P* = 0.09; Figure 2A). There were no significant differences in *R* and *W*_*k*_/*W*_*p*_ between walking conditions and groups (*P* ≥ 0.06). *W*_*p*_*, W*_*kl*_, and β showed a significant interaction effect. *W*_*p*_ was significantly higher in overground than in treadmill walking for both groups (significant walking condition effect; *P* = 0.019; Figure 2B) and in UCP compared with TD on the treadmill (*P* = 0.002). *W*_*kl*_ showed a significant walking condition effect with higher values on the treadmill compared with overground walking (*P* = 0.006; Figure 2D). Moreover, *W*_*kl*_ was significantly higher in UCP than in TD within both walking conditions (*P* < 0.001; Figure 2D). β was significantly higher in UCP compared to TD only on the treadmill (*P* = 0.018).

**Table 5:** **External mechanical work and potential-kinetic energy transduction at preferred walking speed (PWS)**.

**Variable**	**UCP (*****n*** = **9)**		**TD (*****n*** = **10)**		***P*-value**
	**Overground**	**Treadmill**	**Overground**	**Treadmill**	
*W_*ext*_*, J^.^kg^−1.^m^−1^	0.52 ± 0.13	0.49 ± 0.12	0.48 ± 0.16	0.41 ± 0.10	0.36^‡^
*W_*p*_*, J^.^kg^−1.^m^−1^	0.62 ± 0.10	0.61 ± 0.09	0.53 ± 0.12	0.44 ± 0.11	0.049^*^^†^
*W_*k*_*, J^.^kg^−1.^m^−1^	0.76 ± 0.12	0.66 ± 0.09	0.71 ± 0.15	0.61 ± 0.13	0.99^*^
*W_*kf*_*, J^.^kg^−1.^m^−1^	0.74 ± 0.12	0.62 ± 0.09	0.70 ± 0.15	0.60 ± 0.13	0.85^*^
*W_*kv*_*, J^.^kg^−1.^m^−1^	0.11 ± 0.04	0.08 ± 0.04	0.10 ± 0.07	0.05 ± 0.03	0.20^*^
*W_*kl*_*, J^.^kg^−1.^m^−1^	0.03 ± 0.01	0.04 ± 0.01	0.02 ± 0.00	0.02 ± 0.00	0.009^*^^†^
*R*, %	62.9 ± 6.8	61.6 ± 6.6	61.8 ± 6.2	61.3 ± 6.1	0.36
*W_*k*_/W_*p*_*	1.25 ± 0.21	1.11 ± 0.22	1.37 ± 0.22	1.47 ± 0.43	0.07^†^
α, °	18.7 ± 8.4	32.5 ± 12.4	21.3 ± 12.3	28.7 ± 10.6	0.32^*^
β, °	25.6 ± 12.1	29.5 ± 12.6	19.0 ± 9.6	15.6 ± 10.5	0.03^§^

*Mean values ± standard deviation (SD). n, number of participants; UCP, unilateral cerebral palsy adolescents; TD, typically developing adolescents. W_ext_, external mechanical work; W_p_, potential mechanical work; W_k_, kinetic mechanical work; W_kf_, forward kinetic mechanical work; W_kv_, vertical kinetic mechanical work; W_kl_, lateral kinetic mechanical work; R, recovery; α, phase shift between the maximum of E_k_ and the minimum of E_p_; β, phase shift between the minimum of E_k_ and the maximum of E_p_; P-value, P value for interaction [condition (overground vs. treadmill) x group (UCP vs. TD)] of the 2-way repeated-measures mixed design ANOVA*.

* For significant condition (overground vs. treadmill) effect;

† *For significant group (UCP vs. TD) effect (P ≤ 0.05)*.

‡ *For tendency overground vs. treadmill (P = 0.089)*.

§ *For tendency UCP vs. TD (P = 0.053)*.

**Figure 2:** **External (A), potential (B), vertical kinetic (C), lateral kinetic (D) mechanical works at preferred walking speed (PWS)**. UCP, unilateral cerebral palsy adolescents; TD, typically developing adolescents; OG, overground; TM, treadmill; *W*_*ext*_, external mechanical work; *W*_*p*_, potential mechanical work; *W*_*kv*_, vertical kinetic mechanical work; *W*_*kl*_, lateral kinetic mechanical work; ^*^for significant condition (overground vs. treadmill) effect; ^†^for significant group (UCP vs. TD) effect; °For significant interaction (condition × group) effect (*P* ≤ 0.05); ^‡^For tendency overground vs. treadmill (*P* = 0.089).

## Discussion

This study showed that, at SWS, the treadmill compared with the overgound walking induced similar gait mechanical changes in adolescent with UCP (GMFCS level I and II) and TD adolescents, with the exception of *W*_*kl*_ and *W*_*kv*_. Both these kinetic mechanical works were significantly increased during treadmill compared to overground walking only in UCP. In both groups, *W*_*ext*_ was significantly higher on the treadmill compared to overground walking. Contrary to our preliminary hypothesis, the PWS was similar in the two groups in both gait modalities. At this speed, there were similar mechanical changes on treadmill compared to overground walking in adolescents with UCP and TD adolescents, with the exception of *W*_*p*_ and W_*kl*_, confirming the results found for SWS.

### UCP vs. TD adolescents

At SWS in both conditions, there were no differences in spatiotemporal parameters between the two groups except for lateral displacements of COM, which were higher in UCP than in TD in both gait modalities. This finding may attest a larger stride width and greater gait instability in adolescents with UCP as previously suggested by Hsue et al. (2009b). This wide-based gait may be a compensatory strategy for decreasing the activation of weak plantar flexors and hip extensors in UCP (Bennett et al., 2005) associated to lower COM displacements in the forward direction (Hsue et al., 2009b).

At SWS in both gait modalities, *W*_*ext*_ was higher in UCP than in TD. Our findings are in line with studies reporting higher *W*_*ext*_ during overground walking in UCP (Bennett et al., 2005; van den Hecke et al., 2007) and confirm our preliminary hypothesis. The higher *W*_*ext*_ was associated with greater *W*_*p*_, *W*_*kv*_, and *W*_*kl*_ in UCP than in TD. This could be related to the equinus gait pattern common to children and adolescents with CP (Massaad et al., 2004), which affects the COM displacements by increasing the vertical and decreasing the forward displacements. UCP children/adolescents use the vertical stiffness of their paretic lower limb to conserve and release elastic energy during the onset of the stance phase (Fonseca et al., 2004). To optimize this dynamic, adolescents with UCP raise their COM higher than TD adolescents. Our results indicate that higher *W*_*p*_ associated with greater *W*_*kv*_ and *W*_*kl*_ may be an adaptive, compensatory gait mechanism in UCP to optimize the pendular energy transduction, which remains similar in both groups during overground and treadmill walking at SWS. In fact, the higher *W*_*kv*_ and *W*_*kl*_ allow UCP adolescents to increase *W*_*k*_ and, concomitant with the greater *W*_*p*_, to optimize the relative magnitude of *E*_*k*_ and *E*_*p*_ (the ratio *W*_*k*_/*W*_*p*_ was significantly lower and close to 1 in UCP as compared to TD adolescents). The optimization of this relative amplitude compensates the greater phase shift between *E*_*k*_ and *E*_*p*_ (β) and improves *R* up to values similar to TD in adolescents with UCP. Therefore, raising the COM higher onto a plantar flexed foot would present some biomechanical advantages (i.e., conserve and release elastic energy and improve pendular energy transduction) but it may also be a compensatory mechanism for clearing the swing limb. Raising the COM may represent a necessity and specificity of children/adolescents with UCP (Massaad et al., 2004).

At similar PWS in both gait modalities, the two groups walked with similar spatiotemporal parameters. Only the higher lateral COM displacements, *W*_*p*_ and *W*_*kl*_ values characterize the gait pattern of UCP with respect to the one of TD adolescents at this speed, confirming the differences highlighted at SWS. The similar PWS between the two groups is in line with previous studies (Fonseca et al., 2004) and in contrast with others (van den Hecke et al., 2007; van der Krogt et al., 2014, 2015). The low spasticity level and functional limitations of our participants may explain our results. In fact, it has been reported that walking speed and step length were inversely related to spasticity level and force of ankle plantar flexors (Crosbie et al., 2012).

### Overground vs. treadmill walking

At SWS, for both groups, our results showed that the step frequency was higher (6–7%) and the stride duration and length were shorter (6–8%) when walking on the treadmill. This is in line with previous results in adults and children (Stolze et al., 1997; Warabi et al., 2005; Lee and Hidler, 2008). In healthy individuals, it has been suggested that spatiotemporal differences between treadmill and overground may result from the moving belt pulling the stance limb back, thereby inducing an early transition into swing to avoid excessive anterior displacement of the COM (Harris-Love et al., 2001; Brouwer et al., 2009). Reduced knee and hip extension during the push-off phase on the treadmill, explains the reduced stride length and increased stride frequency in order to follow treadmill speed (Murray et al., 1985). In our study the treadmill, reducing lateral COM displacements, decreased gait instability compared to overground walking in both groups. This is in line with previous results reporting decreased stance time variability during treadmill compared with overground walking at the same speed in adults (Warabi et al., 2005). Treadmill locomotion at imposed speed may reduce the possibility of free regulation and induce a constant rhythm with a more symmetric gait pattern (Brouwer et al., 2009).

At SWS, our results showed that *W*_*ext*_ was higher on the treadmill compared to overground walking in both groups. Moreover, concomitant with *W*_*ext*_, *R* was lower with a greater non-significant phase shift between mechanical energies when walking on the treadmill, confirming previous results in healthy adults (Collett et al., 2007). These authors showed a reduced recovery on the treadmill due to greater phase shift between *E*_*k*_ and *E*_*p*_ compared with overground walking. When the COM is behind the foot in contact with the belt, the COM accelerates as it is vertically displaced whereas the treadmill moves the foot backward, thereby inducing an increase in *E*_*k*_ concomitant with *E*_*p*_ increase. Then, the COM is decelerated and moved down in order to maintain a constant speed with the treadmill, thus leading *E*_*k*_ and *E*_*p*_ to decrease simultaneously. Another hypothesis may be that treadmill provides some of the energy to raise the COM, creating an energy exchange between the subject and the treadmill (Savelberg et al., 1998). These results may therefore confirm those of van der Krogt et al. (2015) showing a shift from an ankle to a hip strategy, contributing to increase the *W*_*ext*_ in treadmill compared to overground walking in both groups.

Finally at this speed, only adolescents with UCP showed an increased *W*_*kv*_ and *W*_*kl*_ on the treadmill compared with overground walking whereas these variables remained similar in both gait modalities in TD adolescents. It has been previously reported that, at overground PWS, the vertical and lateral displacements of the COM were faster in UCP than in TD (Hsue et al., 2009a). The faster vertical displacements would help adolescents with UCP to create a higher peak force, used for moving forward the COM during walking. Hsue et al. (2009a) suggested that the vertical acceleration of the COM reflects the capacity of the subject to control external forces (gravity force) and this vertical acceleration would be an index of the postural capacity to control the gravity force. This could reflect the difficulty in UCP to absorb shock as a result of muscular impairments, weakness and stiffness. It is possible that the treadmill accentuates the vertical velocity of the COM and that adolescents with UCP have more difficulties in speed control due to gravity. Therefore, adolescents with UCP would have a reduced adaptive capacity compared to TD adolescents, who absorb and decelerate the speed created by the treadmill better.

The PWS was slower on the treadmill compared to overground walking in both groups. This confirms the findings of many other studies (Hesse et al., 1999; Matsuno et al., 2010; van der Krogt et al., 2014); and may reflect unease associated with treadmill walking (Warabi et al., 2005). A treadmill may generate a discomfort because of the moving belt, since the body is walking but does not move forward. Especially for young subjects, this creates an inadequacy between sensory proprioceptive and visual efferents and affects stability, balance, and perception of body position and walking speed on a treadmill (Stolze et al., 1997). In our study at PWS the transition from overground walking to the treadmill induced almost similar mechanical changes in both groups, and these changes were mainly associated with the slower walking speed on the treadmill. Interestingly, despite the difference in walking speed between the two gait modalities, *R* was similar. Therefore, the two groups chose a PWS which allowed them to optimize pendular energy transduction in both gait modalities. However, as at SWS, the different changes in *W*_*p*_ and *W*_*kl*_ induced by the overground-treadmill transition in the two groups characterize the specific adaptation of the gait pattern of adolescents with UCP. These results confirm the mechanisms previously mentioned to explain the specific gait pattern of UCP compared with TD and the specific adjustments during overground-treadmill transition at SWS in UCP.

### Methodological limitations

Some methodological limitations arose from the study and need to be further addressed. Firstly, *W*_*ext*_ can only account for a fraction of the total mechanical work during walking (i.e., 60–75% in humans, Cavagna and Kaneko, 1977; Russell et al., 2011). Future research should examine *W*_*int*_ to better investigate the biomechanical gait changes during treadmill compared to overground walking in adolescents with CP. Secondly, the use of the displacements of a single anatomical point in children to quantify COM motion may represent a methodological limitation of our study. However, in a previous study (Eames et al., 1999) there was no actual difference between the excursion of a single anatomical point and COM during normal and pathological gait in children. Moreover, *W*_*ext*_ was significantly correlated between the two methods in further studies (Meichtry et al., 2007; Yang and Pai, 2014) and our two groups were compared using the same methodology, which has already been used in adults (Malatesta et al., 2009, 2013) and children (Peyrot et al., 2009, 2010). In contrast to the reference methods usually used to obtain the COM motion (anthropometric modeling and kinematic analysis and ground reaction forces), our method is simple, cheap, consumes little time, and allows clinicians to easily assess the mechanics of overground and treadmill walking in a normal corridor and with a normal treadmill respectively. Therefore, as previously suggested, “the benefits from the simplicity appear to overweigh the limitations in accuracy” (Yang and Pai, 2014). Thirdly, it has recently been shown (Donelan et al., 2002b) that the combined limbs method, used in this study, neglects the work performed during double support stance (*W*_*int, dc*_; Bastien et al., 2003) and thus underestimates the *W*_*ext*_ required to walk. However, Kurz et al. (2010) have recently shown that *W*_*ext*_ was greater than *W*_*int, dc*_ in children with bilateral CP, and that only the former was significantly higher in bilateral CP compared with TD. This attests the relevance of assessing *W*_*ext*_ using the combined limbs method in our population. Finally, the inertial sensors used in this investigation to calculate the spatiotemporal parameters and mechanical work during walking cannot detect the asymmetric influence of the affected and unaffected side on the gait mechanics. However, as already stated in the Methods, GMFCS level I and II unilateral CP adolescents have very limited neuromuscular impairments that affect the symmetry of their gait pattern (Lundh et al., 2014) and limit their mobility. Therefore, our results should be considered specific to adolescents with UCP of these GMFCS levels and should not be extended to adolescents with spastic CP and higher GMFCS levels.

## Conclusions and clinical implications

This study showed that the treadmill compared with overground walking generated similar changes in gait mechanics in adolescents with UCP (GMFCS level I and II) and TD adolescents. However, some specific aspects of the gait pattern of UCP are accentuated during treadmill walking. The overground-treadmill transition induced an increase in *W*_*p*_, *W*_*kv*_, and *W*_*kl*_ only in adolescents with UCP. These results showed that, during treadmill walking, the equinus gait pattern characteristic of these adolescents may be amplified and that UCP reduces the adaptive capacity to absorb and decelerate the speed created by treadmill (i.e., dynamic instability). Dynamic instability, generated by the treadmill, could be used to specifically train the gait pattern and gait stability of adolescents with UCP (GMFCS level I and II). On the other hand, this “artificial” accentuation of some specific aspects of the gait pattern of UCP induced by treadmill walking should be taken into account, when comparing their gait patterns with those of TD adolescents on a treadmill.

## Authors contributions

Conceived and designed the experiments: FD, NP, CN, DM. Performed the experiments: MZ, GC, LP. Analyzed the data: MZ, GC, NP, DM. Interpreted results of research: MZ, FD, GC, LP, NP, CN, DM. Wrote the paper: MZ, DM. Involved in the editing process of the manuscript: MZ, FD, GC, LP, NP, CN, DM.

### Conflict of interest statement

The authors declare that the research was conducted in the absence of any commercial or financial relationships that could be construed as a potential conflict of interest.

## Abbreviations

COM: Center of mass of the human body
CP: Cerebral Palsy
GMFCS: Gross motor function classification system
UCP: Unilateral cerebral palsy
PWS: Preferred walking speed
R: Recovery
TD: Typical development
*W*_*ext*_: External mechanical work
*W*_*int*_: Internal mechanical work
*W*_*k*_: Kinetic mechanical work
*W*_*kf*_: Forward kinetic mechanical work
*W*_*kl*_: Lateral kinetic mechanical work
*W*_*kv*_: Vertical kinetic mechanical work
*W*_*p*_: Potential mechanical work
*W*_*tot*_: Total mechanical work
*α*: Phase shift between the maximum of *E*_*k*_ and the minimum of *E*_*p*_
β: Phase shift between the minimum of *E*_*k*_ and the maximum of *E*_*p*_
SWS: standard walking speed.
